# Identification of Hub Genes in Tuberculosis via Bioinformatics Analysis

**DOI:** 10.1155/2021/8159879

**Published:** 2021-10-11

**Authors:** Tiancheng Zhang, Guihua Rao, Xiwen Gao

**Affiliations:** ^1^Medical College of Soochow University, Soochow University, 199 Renai Road, Suzhou 215123, China; ^2^Department of Laboratory Medicine, Minhang Hospital, Fudan University, China; ^3^Department of Respiratory Medicine, Minhang Hospital, Fudan University, China

## Abstract

**Background:**

Tuberculosis (TB) is a serious chronic bacterial infection caused by Mycobacterium tuberculosis (MTB). It is one of the deadliest diseases in the world and a heavy burden for people all over the world. However, the hub genes involved in the host response remain largely unclear.

**Methods:**

The data set GSE11199 was studied to clarify the potential gene network and signal transduction pathway in TB. The subjects were divided into latent tuberculosis and pulmonary tuberculosis, and the distribution of differentially expressed genes (DEGs) was analyzed between them using GEO2R. We verified the enriched process and pathway of DEGs by making use of the Kyoto Encyclopedia of Genes and Genomes (KEGG) and Gene Ontology (GO). The construction of protein-protein interaction (PPI) network of DEGs was achieved through making use of the Search Tool for the Retrieval of Interacting Genes (STRING), aiming at identifying hub genes. Then, the hub gene expression level in latent and pulmonary tuberculosis was verified by a boxplot. Finally, through making use of Gene Set Enrichment Analysis (GSEA), we further analyzed the pathways related to DEGs in the data set GSE11199 to show the changing pattern between latent and pulmonary tuberculosis.

**Results:**

We identified 98 DEGs in total in the data set GSE11199, 91 genes upregulated and 7 genes downregulated included. The enrichment of GO and KEGG pathways demonstrated that upregulated DEGs were mainly abundant in cytokine-mediated signaling pathway, response to interferon-gamma, endoplasmic reticulum lumen, beta-galactosidase activity, measles, JAK-STAT signaling pathway, cytokine-cytokine receptor interaction, etc. Based on the PPI network, we obtained 4 hub genes with a higher degree, namely, CTLA4, GZMB, GZMA, and PRF1. The box plot showed that these 4 hub gene expression levels in the pulmonary tuberculosis group were higher than those in the latent group. Finally, through Gene Set Enrichment Analysis (GSEA), it was concluded that DEGs were largely associated with proteasome and primary immunodeficiency.

**Conclusions:**

This study reveals the coordination of pathogenic genes during TB infection and offers the diagnosis of TB a promising genome. These hub genes also provide new directions for the development of latent molecular targets for TB treatment.

## 1. Background

Tuberculosis (TB) is a serious chronic bacterial infection caused by Mycobacterium tuberculosis (MTB), which is mainly spread by droplets [1]. It is one of the deadliest diseases in the world and a heavy burden for people all over the world. Its existence not only divides the microorganisms but also causes lung tissue infection [2, 3]. In addition, most patients will have typical symptoms like a low-grade fever, night sweats, and fatigue [4]. TB is difficult to diagnose through clinical, radiology, bacteriology, and histology [5]. Drug treatment is the most important means to treat TB [6], but there are too many patients with drug resistance, especially multiple and extensive drug resistance [7]. So, finding a new way to treat TB is still important.

Currently, the advents of high-throughput sequencing, genomics, and transcriptomics have offered many new remedies for TB treatment [8]. For example, the report by Mboowa et al. mentions that high-throughput sequencing has a wide range of applications in the research of infectious diseases [9]. This technology has generated a large amount of unprecedented information in the history of biology and changed the management of infectious diseases. Chiner-Oms et al. reveal the evolution of the Mycobacterium tuberculosis complex through a large amount of genomics data and find more subtle differences in different human tuberculosis isolates, contributing to the understanding of pathogens and determining the relevant biomedical goals [10]. In addition, van Rensburg and Loxton's research shows that the combined application of transcription pathways and gene expression technologies can help clarify more effective diagnosis and treatment of TB, as well as the development of more effective drug therapies and new vaccines [11]. The identification of biomarkers through transcription profiles can help improve the diagnosis and treatment of TB [12]. The above methods occupy an important position in the research of TB and have been practiced and confirmed by a large number of researchers, which has promoted the diagnosis, cognition, and treatment of TB.

In this research, we analyzed 8 latent tuberculosis and 8 pulmonary tuberculosis samples in the GSE11199 database and then identified differentially expressed genes (DEGs) through GEO2R. Afterward, DEGs were enriched by the Kyoto Encyclopedia of Genes and Genomes (KEGG) and Gene Ontology (GO), and we constructed a protein-protein interaction (PPI) network to identify the hub gene. Finally, we got the key pathways through Gene Set Enrichment Analysis (GSEA). Through the above research, the diagnostic characteristics of TB are explored and the clinical treatment biomarker is found.

## 2. Material and Methods

### 2.1. Gene Expression Microarray Data Acquisition

As a common functional genomics database, the NCBI Gene Expression Omnibus database (GEO, http://www.ncbi.nlm.nih.gov/geo) has high-throughput gene expression sequencing data and microarray data. The gene expression data set GSE11199 [13] was downloaded from GEO. In this data set, 8 pairs of latent tuberculosis and pulmonary tuberculosis samples were analyzed.

### 2.2. Identification of Differentially Expressed Genes (DEGs)

We used GEO2R [14] (http://www.ncbi.nlm.nih.gov/geo/geo2r), a GEO database interactive analysis tool based on the R language, to perform identification of DEG analysis. The genes with log_2_ | fold change (FC) | >1 were defined as differentially expressed. At the same time, with the adjusted*P*value < 0.05, the difference had statistical significance. In addition, we used the volcano to display the latent and pulmonary samples to show the visual hierarchical clustering using ImageGP (http://www.ehbio.com/ImageGP/index.php/Home/Index/index.html).

### 2.3. KEGG and GO Enrichment Analysis of DEGs

Aiming at understanding the function of DEGs, we performed the enrichment analysis by GO and KEGG. The GO and KEGG enrichment in the Database for Annotation, Visualization and Integrated Discovery website (DAVID, https://david.ncifcrf.gov/) was used. GO pathway includes three parts: molecular function (MF), cellular component (CC), and biological process (BP). As a database integrating chemical, genomic, and system function information, KEGG has powerful graphics functions. It shows the metabolic pathways associated with the gene list, which facilitates a comprehensive understanding of the disease.

### 2.4. PPI Network Construction

In order to identify the hub gene of TB patients, we constructed a PPI network by making use of the online database Search Tool for the Retrieval of Interacting Genes (STRING, http://string-db.org). On this basis, the interaction between genes was visualized and the hub genes were predicted according to the strength of the association.

### 2.5. GSEA

According to the GSE11199 data set, TB patients were divided into 8 groups of latent tuberculosis and 8 groups of pulmonary tuberculosis. Aiming at determining the potential functions of DEGs, GSEA on GSE11199 was performed using GSEA 3.0 (http://www.broad.mit.edu/gsea/), and *P* < 0.05 was regarded as statistically significant.

## 3. Results

### 3.1. Identification of DEGs

We downloaded the gene expression profile of GSE11199 from the GEO database, including 2 groups (8 latent tuberculosis subjects and 8 pulmonary tuberculosis subjects). Afterward, we identified 98 DEGs from the GSE11199 data set, including 91 genes upregulated and 7 genes downregulated. We showed the distribution of all DEGs through the volcano graph (Figure 1). The top 7 upregulated genes included MMP12, TACSTD2, IDO1, CCL23, LIMK2, CYP27B1, and CD1B. The top 7 downregulated genes included KITLG, SRPX, HS3ST2, EDNRB, HNRNPU-AS1, HAMP, and CDC42EP3.

### 3.2. GO and KEGG Pathway Enrichment Analysis

GO analysis results demonstrated that in BP, upregulated DEGs were abundant in cytokine-mediated signaling pathway, response to interferon-gamma, peptidyl-tyrosine autophosphorylation, enzyme-linked receptor protein signaling pathway, and other processes. In CC, upregulated DEGs were abundant in endoplasmic reticulum lumen, spindle pole, spindle pole centrosome, and so on. In MF, upregulated DEGs were abundant in beta-galactosidase activity, histone threonine kinase activity, galactosidase activity, etc. (Figure 2(a)). In addition, in the results of KEGG analysis, upregulated DEGs were significantly enriched in the JAK-STAT signaling pathway, cytokine-cytokine receptor interaction, measles, apoptosis, Epstein-Barr virus infection, cell cycle, and other pathways (Figure 2(b)).

### 3.3. PPI Network Construction

Data from the STRING database showed the interaction of given genes. The PPI network of upregulated DEGs consisted of 89 nodes and 96 edges (Figure 3). Among these nodes, with degree ≥ 9 as the screening criterion, the 4 most significant pivot node genes were screened out. These genes were CTLA4, GZMB, GZMA, and PRF1. Among these 4 genes, CTLA4 had the highest node degree (degree = 16), and PRF1 had the lowest node degree (degree = 9). Besides, the expression of these 4 genes was analyzed (Figures 4(a)–4(d)), demonstrating that the expression levels of CTLA4, GZMB, GZMA, and PRF1 in the pulmonary tuberculosis samples were significantly higher than those in the latent control group.

### 3.4. GSEA

The GO and KEGG pathway enrichment analysis was only used to detect DEGs, while the GSEA was used to detect all genes in the data set, which is convenient to supplement other related enrichment pathways. According to Figure 5(a), it could be seen that these genes are significantly enriched in the proteasome pathway, and the normalized enrichment score was 2.353477. The other enrichment pathway was primary immunodeficiency (Figure 5(b)), and its normalized enrichment score was 2.187469.

## 4. Discussion

TB is one of the infectious diseases leading to an increase in morbidity and mortality worldwide [15]. Despite joint efforts to develop new diagnostic methods, drugs, and vaccines and expand pipelines over the past 20 years [16], TB remains a global emergency [17]. In this research, we analyzed the data set GSE11199 in the GEO database to identify the key pathways and hub genes associated with TB. Through the GSE11199 data set, 98 DEGs were identified between latent and pulmonary tuberculosis samples. Among them, the volcano map visually displayed 91 upregulated genes and 7 downregulated genes. Then, according to the GO and KEGG analysis, we obtained the biological processes and pathways associated with upregulated DEGs. The top significantly enriched terms were cytokine-mediated signaling pathway [18], response to interferon-gamma [19], peptidyl-tyrosine autophosphorylation, measles, JAK-STAT signaling pathway [20], cytokine-cytokine receptor interaction [21], Th17 cell differentiation [22], etc. Pai and Rodrigues explain the indirect signs of MTB exposure by interferon-gamma release assay, indicating that there is a cellular immune response to MTB [23]. Studies have shown that Th17 cell differentiation induces neutrophil inflammation, mediates tissue damage, and participates in the pathology of TB [24]. It plays a protective role in the early stage of TB but induces the development of the disease in the late stage of TB.

A PPI network was established using the STRING database, and four hub genes, namely, CTLA4, GZMB, GZMA, and PRF1, were identified through degree value. Therefore, we concluded that these four genes might be related to the onset and treatment of tuberculosis. And these four genes were reported to participate in the development of other diseases. For instance, Froelich J et al. conduct a special study on GZMA in the report, pointing out that GZMA is the most abundant serine protease in killing cytotoxic particles, which activates a new cell death pathway and generates reactive oxygen species in the process [25]. This leads to damage to activated single-stranded DNA, activates monocytes, and produces inflammatory cytokines. Turner et al. confirm that the level of GZMB in chronic diseases and inflammatory skin diseases is significantly higher than the expression level in normal healthy humans and related to skin damage, inflammation, and repair [26]. For CTLA4, Buchbinder and Desai propose in the article that CTLA4 is a negative regulator of T cell immune function and participates in all aspects of immunotherapy for melanoma, non-small-cell lung cancer, and other cancers [27]. In addition, there are few research reports on PRF1, but studies have shown that this gene is involved in expression in diseases such as familial hemophagocytic lymphohistiocytosis type 2 [28], aplastic anemia [29], diabetes, multiple sclerosis [30], and lymphoma [31].

According to the results of GSEA, we found that TB was significantly associated with proteasome and primary immunodeficiency. The study by Samanovic et al. mentions that proteasomes mainly exist in archaea and eukaryotes and are closely related to the pathogenesis of MTB [32]. The occurrence of TB depends on the function of the proteasome, and the biochemistry of the MTB proteasome and its role in virulence are described. Not only that, but Cerda-Maira and Darwin also show in their studies that the proteasome takes responsibility for the degradation of targeted proteins in eukaryotes, and a series of data have also confirmed that the proteasome is related to the pathogenesis of MTB [33]. Glanzmann et al. explain the relationship between individual primary immunodeficiency and TB and, based on survey data in Africa, find that individual loss of primary immune function is more likely to cause TB and other major diseases [34]. This study has some limitations. First of all, the expression level of DEGs needs to be verified by qRT-PCR. Secondly, the specific mechanism of the hub gene in TB needs to be further explored.

In short, we have screed out 98 DEGs, including 91 upregulated and 7 downregulated ones between latent tuberculosis and pulmonary tuberculosis subjects. Then, we get the pathway such as response to interferon-gamma, Th17 cell differentiation, proteasome, and primary immunodeficiency which is largely associated with TB through KEGG, GO, and GSEA. Finally, we identify 4 hub genes through the PPI network; these hub genes could act as biomarkers for the diagnosis or prognosis of TB, providing new directions and technologies for the treatment of TB.

## Figures and Tables

**Figure 1:** The volcano map shows the distribution of DEGs. Based on the GSE11199 database, 98 DEGs were screened out, including 91 upregulated DEGs and 7 downregulated DEGs. Red stands for upregulated genes; blue stands for downregulated genes.

**Figure 2:** GO functional and KEGG pathway analysis of upregulated DEGs. (a) GO term enrichment analysis. The *x*-axis represents enriched GO term description, and the *y*-axis stands for the −log_10_ (*P* value). (b) KEGG pathway enrichment analysis. The colors of the dots represent the *P* values of enrichment, and the size of the dots represents the number of enriched genes.

**Figure 3:** The PPI network of upregulated DEGs. The PPI network is constructed based on the STRING database, and 4 hub genes are screened out.

**Figure 4:** The expression level of the hub gene in the data set GSE11199. The expression level of CTLA4 (a), GZMB (b), GZMA (c), and PRF1 (d) in the latent and pulmonary tuberculosis subjects.

**Figure 5:** GSEA for the KEGG pathway related with tuberculosis based on data set GSE11199. The gene sets of (a) proteasome and (b) primary immunodeficiency were significantly enriched in pulmonary tuberculosis subjects.

## Data Availability

All data analyzed during this study are obtained from a published article or are available from the corresponding author on reasonable request.
